# Optical Coherence Tomography Combined with Fluorescein Fundus Angiography under Intelligent Algorithm to Evaluate the Clinical Efficacy of Ranibizumab Combined with Panretinal Photocoagulation in the Treatment of Macular Edema of Diabetic Retinopathy Patients

**DOI:** 10.1155/2022/2933663

**Published:** 2022-05-02

**Authors:** Ling Li, Qing Zhou, Jing Huang

**Affiliations:** Department of Ophthalmology, The Changsha Fourth Hospital (Affiliated Hospital of Medical College of Hunan Normal University), Changsha, 410006 Hunan, China

## Abstract

This study aimed at investigating the clinical effect of ranibizumab combined with panretinal photocoagulation in the treatment of macular edema in diabetic retinopathy (DR) patients. A parametric deformation model was constructed, and based on this, it was evaluated using optical coherence tomography (OCT) combined with fluorescein fundus angiography (FFA). 56 DR patients (80 eyes) who needed surgery were selected for OCT and FFA scanning, and 0.5 mg ranibizumab was administered intravitreal injection before surgery. It should observe the OCT and FFA image characteristics of patients. In addition, the vision correction status before the surgery, 1 month, 3 months, and 6 months after the surgery, the thickness of the macular retina, operation time, the number of intraoperative electrocoagulation, and complications of patients were recorded. It was found that 82.85% of patients had improved visual acuity after surgery. Compared with preoperative, the average logarithm of the minimum angle of resolution (logMAR) of patients at 6 months after surgery increased significantly (*P* < 0.01). With the increase of the grade of fibrosis and the grade of hemorrhage, the logMAR visual acuity recovery at 6 months after the surgery became worse; the macular retinal thickness at 6 months after the surgery decreased significantly (*P* < 0.01). With the increase of the grade of fibrous proliferation and the grade of bleeding, the operation time, the number of electrocoagulation, and the possibility of iatrogenic holes of patient would increase. It can be known that ranibizumab combined with panretinal photocoagulation surgery could not only reduce the macular edema but also effectively reduce the intraoperative bleeding, simplify the removal of proliferative membranes, decrease the number of electrocoagulation, and shorten the operation time, enhancing the visual function of patients.

## 1. Introduction

In recent years, with the development of population aging and changes in people's lifestyles, the incidence of diabetes in the population has been on the rise. The prevalence of diabetes in the world is about 7.2%, while the prevalence of diabetes in China is about 11.6%, that is, China has more than 100 million diabetic patients, ranking first in the world [1]. Statistics show that by 2030, the number of diabetes patients worldwide is expected to rise from 366 million to 552 million [2]. Therefore, diabetes has become one of the most common chronic diseases that affect people's health. However, if diabetic patients have been ill for a long time, fundus disease, namely, diabetic retinopathy (DR), will occur. Data shows that the incidence of DR in patients with diabetes for more than 30 years exceeds 70% [3, 4].

There are two types of DR, nonproliferative DR (NPDR) and proliferative DR (PDR) [5]. In the early stage of onset, DR is mainly characterized by nonproliferative changes, that is, retinal microaneurysms, hemorrhage, beaded veins, microvascular changes, hard exudation, cotton wool-like plaques, and other changes. If the disease progresses further, it will be characterized by proliferative changes [6]. Relevant studies have pointed out that the incidence of PDR in patients with type 1 diabetes who have been ill for more than 25 years is about 42.9%. At this time, there may be angiogenesis in the retina, which can cause changes in vitreous hemorrhage, fibrovascular membrane formation, and retinal detachment, which requires panretinal photocoagulation treatment [7]. However, because PDR patients often have vitreous hemorrhage, proliferative membranes are drawn, and rehemorrhage is prone to occur during the operation, which makes the epiretinal membrane adhesion, increasing the difficulty to separate and operate, prolonging the operation process, and reducing the effect. However, injecting antivascular endothelial growth factor (VEGF) into the vitreous can effectively prevent angiogenesis and relieve macular edema. One of the most widely used VEGF drugs in clinical practice is ranibizumab [8]. Ranibizumab is a VEGF receptor inhibitor, which can inhibit vascular endothelial cell proliferation, vascular penetration, and cardiovascular genesis by binding and blocking VEGF receptors, with a good adoption value.

The decline in vision in DR is often caused by macular edema. With the development of science and technology, it is difficult to ignore the status of modern medical imaging technology in clinical diagnosis [9]. Optical coherence tomography (OCT) is another new optical imaging technology developed after X-ray computed tomography (X-CT) and magnetic resonance imaging (MRI); and it can achieve high-resolution, noninvasive tomographic measurement of biological tissues, and has very good application prospects [10]. Today, OCT technology has been used in the treatment of many diseases in the clinic, especially for the treatment of ophthalmic diseases. It can observe and quantitatively analyze the ultrastructure in the retina, which has very special significance for the detection and prognosis of the disease in the occurrence and development of DR [11]. Studies have shown that there is a linear regression relationship between the macular thickness measured by the OCT technique and the best-corrected visual acuity, but it cannot completely replace the traditional fundus fluorescein angiography (FFA) [12].

Image segmentation algorithms are usually classified into two categories: voxel-based segmentation and model-based segmentation. The latter can be divided into geometric deformation models and parametric deformation models [13]. Taking into account the prior shape features of the foveal avascular zone (FAZ) in the OCT and FFA imaging process, and the FAZ detection algorithm during the research process, high robustness, and high accuracy is required. Therefore, a topology with faster calculation speed and constant boundary curve was selected in this study. Using specific features such as the uniformity of the image boundary area, the parametric deformation model can be used to limit the active contour [14]. 56 patients (80 eyes) with diabetic retinopathy were enrolled and treated with an intravitreal injection of ranibizumab. By observing OCT and FFA images of the patients, the visual correction before and after surgery, the thickness of the macular retina, the operation time, the number of electrocoagulation, and complications of the patients were recorded to evaluate the clinical efficacy of ranibizumab combined with panretinal photocoagulation in the treatment of diabetic macular edema. It was hoped to provide help for the selection of clinical treatment for diabetic macular edema.

## 2. Materials and Methods

### 2.1. Research Objects

In this study, 56 patients (80 eyes) who were diagnosed with DR in hospital from May 2018 to July 2020 were selected and received OCT and FFA scans. The patients and their families knew about the study and signed the informed consent form. This study has been approved by the medical ethics committee of the hospital.

Inclusion criteria: (I) patients with complete clinical data, (II) patients who signed the informed consent, (III) patients who had not received other treatments, and (IV) patients who were older than 20 years old.

Exclusion criteria: (I) patients with macular edema caused by the macular anterior membrane, macular degeneration, age-related macular degeneration, central retinal vein occlusion, and retinal photocoagulation surgery; (II) patients with severe heart, liver, and kidney diseases; (III) patients with mental diseases; and (IV) patients with poor compliance.

The general conditions of the patients were shown in Table 1. There was no statistically significant difference in the age, course of disease, and other data of all patients (*P* > 0.05). The patients in this study and their family members had fully understood the situation and signed the informed consent forms.

### 2.2. Grade of DR

DR was graded according to the fibrosis observed during the operation [15], as shown in Table 2. DR was graded according to the hemorrhage that occurred during the surgery [16], as shown in Table 3. The lens core hardness was graded according to the emery level standard (Table 4).

All the above levels strictly followed the level standards of the Chinese Medical Association (CMA) Fundus Disease Group in 1985 [17].

### 2.3. Research Methods

- Intravitreal injection of ranibizumab

From the 3rd day before the surgery, local antibiotic eye drops were injected into the diseased eyes, with one drop each time and four times a day. Before the surgery, the eye was rinsed to be operated with iodophor solution, and a suitable position (usually located above the temporal) was selected. The needle tube was inserted vertically into the corneoscleral edge 3.5 mm behind to inject 0.5 mg (0.05 mL) of ranibizumab, and then quickly removed. A medical cotton swab was adopted to compress the bleeding, then, the ofloxacin ointment was applied to the affected eye. The eye was performed with bandage treatment, which should be demolished on the second day.

(II) Design on fully automatic FAZ detection algorithm

There were three main steps for the algorithm: the estimation of the initial search limited of the generalized gradient vector flow (GGVF) of the active contour model ⟶ the generation of the edge map ⟶ the operation. The flow chart was shown in Figure 1.

In the above figure, ①: area growth; ②: morphological operation; ③: geometric center position; ④: finding the largest tangent circle; ⑤: normalization; ⑥: N type OTSU threshold method; ⑦: denoising; and ⑧: GGVF active contour model.

(III) GGVF parametric deformation model

The third step of the FAZ automatic detection algorithm was to run the GGVF active contour model. Through the preprocessing of the first two steps, the initial contour curve and the binary edge image of the GGVF Snake model were experimentally obtained. In the third step, the first two steps were used as the initial input of the GGVF Snake model and started to run to obtain the FAZ area detection result.

The active contour model of Snake was represented by *X*(*k*) = [*x*(*k*), *y*(*k*)], and the evolution function of GGVF Snake model was shown in the following equation:

(1) $$\begin{array}{c} X_{i}\left(k,i\right)=X_{i-1}-\tau \left\{\left(k,i\right)\left[\alpha \frac{\partial^{2}x_{i-1}}{\partial k^{2}}\left(k,i\right)+\beta \frac{\partial^{4}x_{i-1}}{\partial k^{2}}\left(k,i\right)\right]-w\right\}. \end{array}$$

*x*(*k*) and *y*(*k*) referred to the coordinate (*x*, *y*) of the path of the active contour, *k* represented the normalization coefficient of the coordinate point, *τ* represented the evolution step length, and *W*_GGVF_ referred to the external force of the active contour model. At this time, equation below could be obtained:

(2) $$\begin{array}{c} W_{\text{GGVF}}=\iint \left|m\left(\left|\nabla \left.l\right|\right.\right)\right.{\left|\nabla w\right|}^{2}-n\left(\left|\nabla \left.l\right|\right.\right)\left(\left|w-\nabla {\left.l\right|}^{2}\right.\right)dxdy. \end{array}$$

*l*(*x*, *y*) referred to the edge graph, ∇^2^ = *∂*^2^/*∂x*^2^ + *∂*^2^/*∂y*^2^ represented the Laplacian operator, *m*(|∇*l*|) = *e*^−|∇*l*|/*D*^ and *n*(|∇*l*|) = 1 − *m*(|∇*l*|). *m*(|∇*l*|) was adopted to control the tension of the active contour, and *n*(|∇*l*|) was to control the rigidity of the active contour.

### 2.4. Statistical Analysis

All data in the experiment were statistically analyzed by SPSS 19.0 software, and the measurement data were expressed as mean ± standard deviation. Preoperative and postoperative conditions (visual acuity, central retinal thickness of the macula, etc.) were compared using paired *t* test; count data were compared with *χ*^2^ test. When *P* < 0.05, the difference was statistically significant.

## 3. Results

### 3.1. Thickness of Macular Retina

80 eyes were examined by FFA, 60 eyes (75%) were diagnosed with diabetic macular edema, and 20 eyes (25%) were not found to have the diabetic macular edema. After OCT examination, 8 eyes (10%) were not found with thickened macular retinal, and 72 eyes (90%) were found with thickened macular retinal. The details were shown in Figure 2, Table 5, and Figure 3.

Figure 2(a) was a normal retina, Figure 2(b) was a nonproliferative DR, Figure 2(c) showed a proliferative DR, Figures 2(d) and 2(e) were segmented images of diabetic macular edema in fundus OCT images, and Figure 2(f) was an OCT of cystoid macular edema image.

The changes in the data in Table 5 and Figure 3 revealed the *χ*^2^ test that the sensitivity of OCT inspection was much greater than that of FFA inspection (*P* < 0.01), and the difference was statistically significant.

The macular retina thickness values measured by the patients before and after the surgery in this study were shown in Figure 4. As illustrated in Figure 4, the thickness of macular retina at 6 months after surgery was significantly decreased compared with that before surgery (*t* = 6.93, *P* ≤ 0.001), and the difference was statistically significant.

### 3.2. Visual Acuity

In this study, the preoperative and postoperative logarithm of the minimum angle of resolution (LogMAR) visual acuity values of all patients in this study were shown in Figure 5. Figure 5 illustrated that compared with preoperative, the patient's average logMAR visual acuity at 6 months postoperatively increased significantly (*t* = 6.11, *P* ≤ 0.001), and the difference was statistically significant.

All patients were stratified according to the classification of fibrosis and hemorrhage, and the level of logMAR visual acuity improved at 6 months after surgery, as shown in Figure 6. As given in Figure 6, as the grade of fibrosis and the grade of hemorrhage increased, the patient's logMAR vision recovery at 6 months after surgery became worse. For the prognosis of patients, fibrosis grading had a greater impact than hemorrhage grading, especially when fibrosis was graded 3, the prognosis was significantly reduced. The visual acuity of all patients at 6 months postoperatively improved at fibrosis level 1; when the fibrosis grade was at level 2, 2 patients had visual acuity at 6 months postoperatively; and when fibrosis was in grade 3, 3 patients had visual acuity loss 6 months after surgery, and 2 patients had no obvious change in visual acuity 6 months after surgery.

### 3.3. Operation Time

The average operation time of all patients in this study was 43.34 ± 16.22 minutes. After stratification according to the classification of fibrosis and hemorrhage, the operation time of all patients was shown in Figure 7.

Figure 7 suggested that as the grade of fibrosis and hemorrhage increased, the operation time of the patient increased, and the degree of influence of fibrosis grading was greater compared with the grade of hemorrhage.

### 3.4. Number of Intraoperative Electrocoagulation

The average number of intraoperative electrocoagulation in all patients in this study was 2.21 ± 0.74 times. After stratification according to the classification of fibrosis and hemorrhage, the number of intraoperative electrocoagulation in all patients was shown in Figure 8.

As Figure 8 illustrated, compared to the fibrosis classification, the hemorrhage classification had a greater impact on the number of intraoperative electrocoagulation, that was to say the number of intraoperative electrocoagulation patients increased as the hemorrhage classification level increased.

### 3.5. Intraocular Pressure

The intraocular pressure values of the patients before and after the surgery in this study were shown in Figure 9.

5 patients had transient high intraocular pressure. The maximum intraocular pressure was 27.42 mmHg. All patients with increased intraocular pressure used eye drops to reduce intraocular pressure. After treatment, the intraocular pressure returned to normal.

### 3.6. Complications

In this study, there were 9 patients with complications of iatrogenic holes. After stratification according to the classification of fibrosis and hemorrhage, the number of concurrent iatrogenic holes was shown in Figure 10.

As Figure 10 showed, compared with the classification of hemorrhage, the classification of fibrosis would have a greater impact on the iatrogenic holes. Therefore, as the classification of fibrosis increased, the probability of patients with iatrogenic holes increased.

## 4. Discussion

Relevant studies have shown that in the diagnosis of macular edema, FFA can accurately locate the vascular leakage and ischemic areas of the macula, but it is difficult to find when there is a very small amount of subretinal fluid [18]. At the same time, the change of retinal thickness in the macular area cannot be quantitatively measured [19]. However, what is really related to the decrease in vision is not the leakage of blood vessels, but the thickness of the retina in the macula. On the contrary, based on the effect of light waves on eye tissues, OCT can perform tomography in different directions and positions and can quantify the structure of the cross-section while displaying the structure. It is possible to observe the slight thickening of macular retina earlier and quantitatively analyze the thickness change before leakage occurs. In addition, its reproducibility, good sensitivity, and strong specificity are noninvasive tests [20]. However, as an indirect measurement method, OCT is easily affected by fixation function and refractive index. Therefore, it cannot completely replace FFA. The application of the two should complement each other.

According to related literature, macular edema images can be manifested in three types: retinal cavernous edema, macular cystic edema, and neuroepithelial serous detachment [21]. In this study, retinal cavernous edema accounted for 37.5%, and macular edema was simpler than typical FFA examination. However, in the event of severe local or diffuse macular leakage, fluorescein may cover the cystic colored image, making the diagnosis neglected. The advantage of OCT is to clearly show the small cyst and indicate the location of the retina. 11 eyes (13.8%) were detected no neuroepithelial serous detachment in FFA examination, which may be able to answer the unexplained decreased vision in diabetic macular disease.

Panretinal laser photocoagulation (PRP) can destroy some relatively hypoxic tissues in the outer layer of the retina and fundamentally reduce the oxygen consumption of the retina, thereby improving the hypoxic condition of the inner layer of the retina. Therefore, it can effectively inhibit the release of some neovascular factors caused by hypoxia, thereby reducing the regeneration of neovascularization [22]. According to this experiment, the thickness of the macular retina decreased significantly 6 months after surgery compared with that before surgery (*t* = 6.93, *P* = 0.000 < 0.01), with statistical differences. It indicated that ranibizumab combined with panretinal photocoagulation could not only effectively improve macular edema but also improve the visual ability of the patient. Some researchers said that in the treatment of PDR with panretinal laser photocoagulation, 66.67% of patients had improved vision after surgery [23]. In this study, after intravitreal injection of ranibizumab was given to patients before PRP surgery, 82.85% of patients had improved vision after surgery, and the effect was better. At the same time, it was found that compared with preoperative PDR patients, the average logMAR visual acuity of patients at 6 months after surgery increased significantly (*P* < 0.01), and the difference was statistically significant. With the increase in the classification of fibrosis and hemorrhage, the patient's logMAR vision recovery at 6 months after the surgery became worse. For the patient's prognosis, fibrosis grading had a greater impact, especially when fibrosis was grade 3, the prognosis was significantly reduced; the thickness of macular retina at 6 months after surgery was significantly reduced (*P* < 0.01), and the difference was statistically significant. As the grade of fibrosis and hemorrhage increased, the patient's operation time increased, and the degree of influence of fibrosis grading was greater. The grade of hemorrhage had a greater impact on the number of intraoperative electrocoagulation, that was, the number of intraoperative electrocoagulation of patients increased as the grade of hemorrhage increased. The degree of fibrosis grading had a greater impact on iatrogenic holes, that was, the possibility of patients with iatrogenic holes increased as the fibrosis grading level increased. It has been reported that intravitreal injection of ranibizumab has a positive effect on the prevention and treatment of hemorrhage after PDR [24]. All patients in this study did not have obvious postoperative complications.

## 5. Conclusion

In this study, the surgical treatment of DR was explored, and the clinical efficacy of ranibizumab combined with panretinal photocoagulation was evaluated by using OCT + FFA based on the parametric deformation model. It was found that the treatment method proposed in this study could not only reduce macular edema but also effectively lessen the hemorrhage during surgery, making it easy to remove proliferative membranes, reducing the number of intraoperative electrocoagulation, shortening the operation time, and significantly improving the visual function of the patient. Nevertheless, due to the small sample content and lack of controlled experiments in this study, the analysis results are not precise enough. Hence, more patients will be included in the subsequent research to further analyze the role of ranibizumab in ophthalmic surgery. In conclusion, the results of this work provided the data reference for the clinical treatment of diabetic macular edema.

## Figures and Tables

**Figure 1:** Flow chart of automatic FAZ detection algorithm.

**Figure 2:** Images of retina ((a)–(c) retinal images; (d)–(f) OCT images).

**Figure 3:** Changes on FAA macular area fluorescence leakage and OCT retinal thickness.

**Figure 4:** The thickness of the macular membrane before and after the surgery (∗# indicated the difference was statistically significant (*P* < 0.01)).

**Figure 5:** LogMAR visual acuity values of patients before and after surgery (∗# meant the difference was statistically significant (*P* < 0.01)).

**Figure 6:** The improved level of logMAR visual acuity of patients in each stratification 6 months after surgery.

**Figure 7:** Operation time of each stratified patient.

**Figure 8:** The number of intraoperative electrocoagulation of each stratified patient.

**Figure 9:** The intraocular pressure of the patient before and after surgery.

**Figure 10:** Number of iatrogenic holes in patients by stratification.

**Table 1:** General data of patients.

Gender	Number of cases	Number of affected eye	Proportion of ill eyes	Age (years old)	Average age	Course of disease
Males	30	38	47.5%	34~80 years old	62.71 years old	5 ~ 34 years
Females	26	42	52.5%			

**Table 2:** Grades based on fibrosis.

Grade	Descriptions
Grade 1	Proliferation confined to the front of the retina (less than 3 locations)
Grade 2	Extensive adhesions occurred in the macula, vascular arch, optic disc, etc., or proliferation spread to the adjacent omentum (at least 1 and less than 3)
Grade 3	Proliferation spread to the adjacent omentum or extensive adhesions (more than 3 locations)

**Table 3:** Grades based on hemorrhage.

Grade	Descriptions
Grade 1	Punctate hemorrhage occurred during the surgery, hemorrhage can be stopped after increasing the intraocular pressure
Grade 2	Diffuse hemorrhage occurred during the surgery, and hemorrhage can be stopped after electrocoagulation
Grade 3	During the surgery, hemorrhage occurred at the posterior part of the fundus and was greater than 1/2, and the hemorrhage could not be coagulated or the operation should be stopped midway

**Table 4:** Emery level standard.

Level	Descriptions
Level I	Transparent color, no core, soft
Level II	Yellowish white or yellow, soft core
Level III	Dark yellow, medium hardness core
Level IV	Brown or amber, hard core
Level V	Tan or black, very hard core

**Table 5:** OCT image display results.

Pathological type	Number of affected eyes	Image characteristics
Retinal spongiform edema	30 (37.5%)	The thickness of the retina increased, the internal reflection decreased, and the low reflection area increased
Macular cystic edema	19 (24.7%)	Vesicle-like changes occurred in the center of the macula, and fluid cavities (various sizes) appeared in the nerve fiber layer
Neuroepithelial serous detachment	11 (13.8%)	There was fluid under the retina and the retinal border detachment was significant

## Data Availability

The data used to support the findings of this study are available from the corresponding author upon request.
